# NT-proBNP Levels and Collateral Circulation Status in Patients with Acute Ischemic Stroke

**DOI:** 10.1155/2023/5318012

**Published:** 2023-04-14

**Authors:** Xiaozhu Shen, Xianxian Zhang, Mengqian Liu, Nan Dong, Juan Liao, Guoqing Zhou, Zhiyong Cao, Liqiang Yu, Yiwen Xu, Yi Jiang, Yue Wan, Qi Fang

**Affiliations:** ^1^Department of Neurology, First Affiliated Hospital of Soochow University, Suzhou, China; ^2^Department of Geriatrics, Lianyungang Second People's Hospital, Lianyungang, China; ^3^Department of Neurology, Yancheng Third People's Hospital, Yancheng, China; ^4^Department of Neurology, Suzhou Industrial Park Xinghai Hospital, Suzhou, China

## Abstract

**Methods:**

In this study, 326 hospitalized patients with acute anterior circulation ischemic stroke (AACIS) were included. A comparison of the clinical characteristics of those with and without AF was conducted. The Spearman rank correlation was used for the correlation analysis of plasma NT-proBNP level, regional leptomeningeal collateral (rLMC) score, and computed tomography perfusion (CTP) status in the AF and non-AF groups. An analysis of multivariate linear regression was used to determine how plasma NT-proBNP level, rLMC score, and CTP status influenced the score on the NIHSS.

**Results:**

There was a greater plasma NT-proBNP level in the AF group compared with the non-AF group, an increased CTP volume (including CTP ischemic volume, CTP infarct core volume, and CTP ischemic penumbra volume (*P* = 0.002)), higher NIHSS score on admission, and lower rLMC score (*P* < 0.001 for the remaining parameters). A negative correlation exists between plasma NT-proBNP level and rLMC score (*r* = −0.156, *P* = 0.022), but a positive correlation exists between plasma NT-proBNP level and both CTP ischemic volume and CTP infarct core volume (*r* = 0.148, *P* = 0.003) in the AF group, but not in the non-AF group. Multivariate linear regression analysis demonstrated that NT-proBNP, CTP ischemic penumbra volume, and rLMC score were associated with NIHSS score, and NT-proBNP was positively associated with NIHSS scores (95% confidence interval (CI), 0.000-0.002; *P* = 0.004) in the AF group, whatever in the unadjusted model or adjusted models, but not in the nonlarge artery atherosclerosis (LAA) group.

**Conclusion:**

In AACIS patients with AF, NT-proBNP level negatively correlated with collateral status, positively with CTP ischemic volume, and positively with NIHSS score.

## 1. Introduction

Every year, China suffers about 3.94 million new stroke cases and a couple of 19 million stroke-related deaths. In 2019, China can have approximately 28 million stroke sufferers, such as 24 million ischemic strokes [1]. The incidence of AF is growing international due to its excessive occurrence within the elderly and the getting older of the global population [2]. In addition to atrial traumatic inflammation, the chance of a cardiac embolic event (CEA) increases extensively with age [3]. CEA is characterised through a big infarct, excessive neurological damage, and a poor analysis. It debts for much less than 30% of all ischemic strokes, while ischemic strokes associated with atrial traumatic inflammation account for approximately 79% of cardiogenic strokes [4, 5].

The natriuretic peptide (NP) circle of relatives is a class of hormones, and their receptors recognized for their useful consequences on the cardiovascular system [6]. Heart patients who suffer from ventricular enlargement or strain overload are secreted B-type natriuretic peptide. A study of sufferers with embolic stroke of undetermined motive (ESUS) discovered that those sufferers had silent AF or were at risk of developing AF after initial evaluation and that advanced age and elevated BNP (NT-proBNP) stages have been considerable independent predictors of AF [7]. In addition, serum NT-proBNP levels can be used as a biological indicator to assess the severity of the stroke [8]. Plasma BNP stages are substantially better in patients with atrial traumatic inflammation than in patients without atrial traumatic inflammation [9]. However, the effects of BNP on stroke have no longer been fully explored.

Previous studies have shown that LAA accidents have a better collateral recruitment than CES [10, 11]. The collateral circulation of the mind, which may be defined as an anastomosis between arteries, can provide nutrient perfusion to areas of the mind in which the main supply of blood flow has been decreased or destroyed through ailment, along with stroke. Collateral stream is every other critical aspect influencing stroke severity and NIHSS score [12]. Therefore, ischemic strokes associated with atrial fibrillation are generally more extreme than those of different aetiologies due to thromboembolic occasions [13].

The rLMC score based totally on CTA photographs was used to assess the collateral circulate. The visibility of collateral circulate on CTA is particularly depending on the time of acquisition. The electricity of the collateral circulation is extra essential for tissue fate than the collateral filling price [14, 15]. The collateral stream is quite variable between individuals, and the optimum time of series is also in my view variable [16]. The CTP generates a couple of maps of ischemic tissue and is a regarded decision-making device for patients with acute ischemic stroke [17]. In addition, CTP is regularly used to useful resource choice making in sufferers with acute ischemic stroke and has been proven to be powerful for not on time remedy (beyond 6 hours) in those patients [18].

To date, few studies have centered at the effect of BNP on collaterals, and we have formerly posted a paper at the affiliation among BNP and stroke outcome [19]. In this study, NT-proBNP levels were evaluated in patients with or without atrial fibrillation to determine how they affect collaterals and to discover the impact of NT-proBNP tiers on CTP imaging and NIHSS rankings in patients with ACIS, as a result supplying a mechanism underlying the effect on stroke severity.

## 2. Methods

### 2.1. Study Population

This study examines statistics for patients admitted to Soochow University's First Affiliated Hospital's Stroke Center from March 2018 to January 2021. As illustrated in Figure 1, the flow diagram illustrates the inclusion and exclusion of affected persons. In total, 326 patients were included in the study. Patients meeting the following criteria were protected: (1) age ≥ 18 years vintage; (2) the onset of AACIS inside 24 h; (3) anterior circulation ischemia, confirmed by imaging (magnetic resonance angiography (MRA) or CT); and (4) the plasma NT-proBNP level will be measured within 0.5 hours of admission to the hospital, along with the current CTA+CTP process. The following standards have been used for exclusions: (1) hemorrhaging or mass in the brain (cerebral hemorrhage was excluded via emergency cranial CT, such as publish-infarction hemorrhage after hospitalization); (2) patients with temporary ischemic assault; (3) patients with severe contamination or septic surprise; (4) patients with history of intense trauma who obtained surgical treatment; (5) obvious liver and renal failure; (6) endocrine, immune, and neoplastic disease; (7) pregnancy; and (8) other causes of cardiogenic stroke (e.g., patent foramen ovale, left atrial myxoma, rheumatic heart disease, dilated cardiomyopathy, and hypertrophic cardiomyopathy). Ethical popularity of this study was acquired from the Ethics Committees of the First Affiliated Hospital of Soochow University (Approval Nos. 2020272 and 2019057).

### 2.2. Data Collection

Prior history of enrolled sufferers protected age, gender, history of smoking, history of high blood pressure, diabetes mellitus, stroke, own family records of stroke, the clinical parameters obtained from the bodily exam, inclusive of peak, weight, frame mass index (BMI), systolic blood pressure (SBP), diastolic blood stress (DBP), blood glucose degree on admission, the NIHSS score, the nearby leptomeningeal collateral (rLMC) rating, and so forth. Hypertension is defined as SBP ≥ 140 mmHg or DBP ≥ 90 mmHg. Diabetes mellitus was described as undergoing remedy with insulin or antidiabetic pills, fasting glucose degree ≥ 7.0 mmol/L, or glycated hemoglobin (HbA1c) ≥ 6.5%. An individual's BMI is calculated by dividing their weight in kilograms by the square of their height in meters. Laboratory checks covered the serum creatinine (Cr), triglycerides (TGs), total LDL cholesterol (TC), low-density lipoprotein LDL cholesterol (LDL-C), excessive-density lipoprotein LDL cholesterol (HDL-C), albumin (ALB), cardiac troponin I (TnI), D-dimer, platelet count number (PLT), global normalized ratio (INR), fibrinogen (FIB), activated partial thromboplastin time (APTT), homocysteine (Hcy), and plasma NT-proBNP.

### 2.3. Treatment

Patients who were suspected of having stroke onset by neurologists (or were visited in good condition) within 24 h were subjected to multimodal CT imaging (noncontrast CT (NCCT)+CTA+CTP). GE Revolution CT (GE Healthcare, Chicago, IL, USA) was used for inspection. The NCCT was acquired with voltage of 120 kV, contemporary of 320 mAs, slice thickness of 0.625 mm, and reconstructed slice thickness of 5 mm. The CTP parameters were voltage of 80 kV and the present day of one hundred fifty mAs. During the intravenous management of 40 mL ioversol (Ultravist 370, Bayer Healthcare, Berlin, Germany), gantry rotations have been constantly executed at a management price of 5 mL/s (every 2 s for 60.Three); after which, 50 mL saline was administered. To perform CTA, patients were intravenously administered with 40 mL ioversol at a flow price of 5 mL/s, accompanied through intravenous administration of 50 mL regular saline. None of the sufferers have been allergic to contrast. The sufferers' remedy decisions (along with intravenous thrombolysis as each fashionable-dose (0.9 mg/kg) thrombolysis and coffee-dose (0.6 mg/kg) thrombolysis and thrombectomy, without inclusion of recanalization remedy) were made with the help of skilled neurologists.

### 2.4. Collateral Flow Imagining

CTP ischemic penumbra quantity was measured to reflect collateral repute. All CTP images have been submitted and processed with the use of the MIStar software (Apollo Medical Imaging Technology, Melbourne, Australia) with single-fee deconvolution and delay and dispersion correction. Previously demonstrated thresholds were carried out to measure the CTP ischemic penumbra quantity (delay time (DT) > 3 s) and CTP infarct core extent (relative cerebral blood flow (rCBF) < 30%). Acute hypoperfused lesions minus infarct center volume were used to calculate CTP ischemic penumbra quantities (Figure 2).

### 2.5. Assessment of Leptomeningeal Collateral Status

By consensus (BKM, SIS), the rLMC rating (20 factors) is used to assess the leptomeningeal collateral reputation based on baseline CTA. RLMC score is based totally on scoring volume of contrast opacification in arteries distal to an M1 MCA/ICA occlusion (0, artery now not visible; 1, less outstanding; and 2, identical or extra outstanding in comparison with a matching region inside the opposite hemisphere) inside the 6 ASPECTS cortical areas (M1-6), parasagittal ACA territory, and basal ganglia. Within the scoring, lenticulostriate arteries arising from retrogradely filled MCAs distant from an occlusion are protected. Arteries inside the Sylvian sulcus are given a better rating, i.e., 0, 2, or 4 (0, now not visible; 2, less; and 4, same or prominent as compared with the alternative Sylvian sulcus) due to the fact that opacification of those vessels maximum remote from leptomeningeal ACA to MCA and PCA to MCA anastomoses is a robust indicator of excellent retrograde waft via those collateral networks. Higher total ratings indicate higher collateral repute. RLMC rating was assessed blinded to clinical information by way of experienced neuroradiologists (ND and JL) for the presence.

### 2.6. Statistical Analysis

All statistics had been analyzed using the SPSS 22.0 (IBM Corp., Armonk, NY, USA) and GraphPad Prism 9.0.0 (GraphPad Software Inc., San Diego, CA, USA) software program. In a tailed test, *P* < 0.05 was taken into consideration as statistically vast.

Patients' baseline characteristics and the single-aspect as stratified via TOAST types were analyzed with the use of the subsequent techniques. Numerical variables are tested for normality using the Kolmogorov-Smirnov test; median and interquartile range (IQR) have been utilized to describe abnormally disbursed nonstop variables. The normally distributed continuous variables were analyzed by the independent sample *t*-test. The data, including PLT and LDL-C, were expressed as mean ± standard deviation (SD). Data that were dispensed abnormally were analyzed by using the Mann–Whitney *U* tests, which include age, SBP, DBP, blood glucose stage on admission, NIHSS score on admission, top, frame weight, BMI, rLMC score, CTP ischemic extent, CTP infarct core quantity, CTP ischemic penumbra extent, NT-proBNP, TnI, D-dimer, INR, FIB, APTT, Cr, TG, TC, HDL-C, ALB, and Hcy. The categorical variables have been expressed as count number and percent, and the Chi-rectangular test or the Fisher's precise test was used for comparing information (gender, records of hypertension, diabetes mellitus, stroke, smoking, and own family history of stroke) between groups (Table 1). The Spearman rank correlation was used for the correlation evaluation of NT-proBNP and rLMC rating, as well as CTP reputation in the AF and non-AF groups (Table 2 and Figure 3).

The influence of NT-proBNP, CTP ischemic penumbra volume, and rLMC score on NT-proBNP was also examined using multivariate linear regression models on NIHSS rating in AF organization (*n* = 113) and non-AF group (*n* = 213), via adjusting the ability confounding clinical variables (Tables 3 and 4). By using the Brant test, the proportionality assumption of the proportional odds model was tested.

## 3. Results

### 3.1. Participants' Clinical Characteristics

Table 1 summarizes members' scientific traits. Compared with the non-AF institution, sufferers in the AF group were older and had higher plasma NT-proBNP degree, larger CTP quantity (such as CTP ischemic quantity, CTP infarct core extent, and CTP ischemic penumbra volume (*P* = 0.002)), higher NIHSS score on admission, and lower rLMC score (*P* < 0.001 for the remaining parameters). In addition, gender, SBP, height, weight, BMI, smoking, TnI level, D-dimer level, INR, APTT, TG level, TC level, and ALB level were also statistically different between the two groups (all *P* < 0.05).

### 3.2. Spearman's Rank Correlation Analysis of NT-proBNP Level, rLMC Score, and CTP Status

Table 2 and Figure 3 show the results of the Spearman rank correlation analysis of plasma NT-proBNP level, rLMC score, and CTP status in the AF and non-AF groups. In the AF group, plasma NT-proBNP level was negatively correlated with rLMC score (*r* = −0.156, *P* = 0.022) (Figure 3(a)), while it was positively correlated with CTP ischemic volume (*r* = 0.137, *P* = 0.045) (Figure 3(b)) and CTP infarct core volume (*r* = 0.148, *P* = 0.003) (Figure 3(c)). However, it was revealed that in the AF group, there was no significant correlation between plasma NT-proBNP level and CTP ischemic penumbra volume (*P* = 0.135 > 0.05) (Figure 3(d)). The correlations among all indices in the non-AF group were not statistically significant.

### 3.3. Multivariate Linear Regression Analysis of the Effects of NT-proBNP, CTP Ischemic Penumbra Volume, and rLMC Score on NIHSS Score in the Two Groups

Tables 3 and 4 show the association of plasma NT-proBNP, CTP ischemic penumbra volume, and rLMC score with NIHSS score in the AF and non-AF groups by the multivariate linear regression analysis.  Table 3 indicates that in the basal unadjusted model (model 0), each 1000-unit increase in plasma NT-proBNP level is associated with a 1-unit increase in NIHSS score (95% confidence interval (CI), 0.000-0.002; *P* = 0.004). After adjusting for the confounding clinical variables in the other models (model 1 and model 2), this correlation can be still confirmed. However, the rLMC score was negatively correlated with the NIHSS score, which was observed in all the three models.

In addition, using multivariate linear regression analysis, as shown in Table 4 (whatever in the unadjusted model or adjusted models), the association between plasma NT-proBNP level and NIHSS score was not found in the non-AF group.

## 4. Discussion

Although CES related to atrial fibrillation has been stated to be associated with ischemic lesions in numerous cerebrovascular areas, preceding research has recommended that CES is related to big infarcts in cerebral arterial areas [20]. This examination confirmed that patients in the atrial fibrillation institution had been older and had better NT-proBNP stages on admission, larger CTP ischemic volumes, larger CTP imperative infarct volumes, and higher NIHSS ratings. This is steady with the characteristics of sufferers with CES associated with atrial fibrillation. This study's results are consistent with those in Zecca and Gutierrez, in which stroke patients with atrial fibrillation had higher NT-proBNP levels and NIHSS scores [21, 22]. Possible motives for the larger CTP volumes in the atrial traumatic inflammation institution can be associated with the usual large infarct length in the atrial fibrillation institution as compared to the nonatrial fibrillation institution, which is likewise related to the better NHISS score [23].

Carotid atherosclerosis has been growing in human beings for many years and is specially followed with the aid of narrowing of the arteries that can sell collateral move inside the brain [24]. In contrast, the prevalence of collateral artery formation and recruitment was decrease in those patients, with CES now not being related to continual cerebral underperfusion [10]. There has been a connection between large infarct length and poor collateral circulation, according to previous studies, perhaps because the presence of a larger penumbra is associated with excellent movement within the collateral pathway, and the time window for possible reperfusion can be extended by prolonging the survival time of the penumbra [25]. According to a study published in 2021, ischemic stroke victims who present within 24 hours of onset have extremely high chances of surviving; the penumbra device permits for secure and effective revascularisation; in other phrases, properly collateral stream limits the enlargement of the infarct core and determines the final infarct volume [16]. Thus, CES related to atrial traumatic inflammation is related to more extreme hypoperfusion, main to larger infarct volumes, extra intense haemorrhagic transformation, and worse stroke outcomes than LAA [26, 27]. Since BNP is considered a marker of cardiogenic stroke (W. [28]) and is associated with collateral circulation formation, which affects the prognosis of cardiogenic stroke, it is possible that our BNP may influence the prognosis of cardiogenic stroke by affecting the collateral circulation.

In the present study, NT-proBNP levels in the AF group were found to be negatively correlated with rLMC scores, whereas NT-proBNP levels in the non-AF group were not correlated with rLMC scores; the explanation for this difference needs further investigation. Furthermore, within the modern-day, have a look at LAA accounted for the majority of instances within the non-AF organization (77.9%). The motive for the lower rLMC rating in the AF organization may be associated with an insufficient opening of the aspect department inside the time window, as it may additionally be legitimate for the non-AF organization to have a better beginning of the side branch just before stroke onset [11, 24]. It has been said that persistent hypoperfusion because of atherosclerotic stenotic lesions effects in higher collateral recruitment as compared to CESs. This might also partly provide an explanation for the poorer final results of AF-related stroke [9]. Another observation confirmed that non-CES patients had particularly higher collateral movement, larger ischemic penumbra volumes, and smaller ischemic middle volumes compared to CES patients [10].

The present look at showed that other risk elements, together with higher systolic blood stress, better TG tiers, higher TC stages and higher ALB ranges, had been chance factors for the improvement of non-FA ischaemic stroke, that is steady with formerly said findings and may be related to their key function inside the pathophysiological pathways worried in atherosclerotic development [29, 30]. Non-AF ischemic stroke was also observed to be related to hazard elements such as gender (male), high BMI, and smoking, which is consistent with preceding findings [31]. In addition, TnI, D-dimer, aPTT, and INR degrees have been higher within the AF organization, that is, regular with preceding studies, as coagulation problems are associated with an excessive hazard of AF [32, 33].

In this study, splendid correlations between NT-proBNP ranges, CTP infarct middle quantity, and CTP ischemic extent in atrial disturbing inflammatory bodies have been decided. The dating among plasma BNP tiers and infarct length (regions of immoderate sign intensity) was studied in 141 sufferers within 3 days of infarct onset with the use of diffusion-weighted imaging (DWI), and an increase in plasma BNP degrees was found to be associated with a boom inside the wide variety of infarcts and with a growth inside the quantity of infarcts [9]. This result is regular with the relationship between plasma BNP tiers and CTP infarct extent inside the atrial fibrillation organization on this study. The nice correlation between infarct volume and plasma BNP tiers might also imply that a capability supply of plasma BNP is the damaged brain.

However, there has been no correlation among NT-proBNP degree, PTC infarct core volume, and PTC ischemic volume in the non-AF organization in the present observation. The actual mechanism of BNP elevation in acute cerebral infarction remains unknown. There is a hypothesis that multiplied BNP in acute cerebral infarction is associated with AF, which may be associated with cardiovascular illnesses associated with AF, or with structural adjustments inside the atrial myocardium, which may be the cause of the cerebral infarction, a coexisting circumstance, or an effect of the cerebral infarction [34, 35]. This may additionally explain why AF-associated stroke is related to higher NT-proBNP tiers, poorer fine facet branches, and larger infarct length.

Since the treatment strategies of AF-related stroke and non-AF-related stroke are not completely constant, we studied the connection among BNP stage and collateral movement as well as whether or not it is far AF-related stroke. This measure can interfere as early as viable in AF-related stroke and thus reduce its mortality and incapacity price.

This is a cross-sectional study; the causal relationship and specific mechanism between BNP and stroke type are still unclear. This is a single-center retrospective study, and there may be a selection bias. The populace of this observe changed into Asian, and the results will not be applicable to different ethnic agencies. In addition, because of the regression analysis, the correlations presented are statistically widespread and their price for the scientific speculation may be uncertain.

## 5. Conclusions

In précis, findings of the contemporary observation indicated that NT-proBNP degree was negatively correlated with collateral repute, while it was undoubtedly correlated with CTP ischemic volume. Besides, NT-proBNP degree was undoubtedly correlated with NIHSS rating in AACIS sufferers with AF. The results suggested that AF-associated stroke was related to a better NT-proBNP level, worse collateralization, and a larger infarct length.

## Figures and Tables

**Figure 1:** Flow diagram of included and excluded patients.

**Figure 2:** MIStar automatic software was used to calculate ischemic volume. CTP ischemic volume (red): DT > 3 s^+^. CTP infarct core volume (green): CBF < 30%. CTP ischemic penumbra volume (green minus red): mismatch: acute hypoperfused lesion volume minus the infarct core volume.

**Figure 3:** Scatter plots illustrating results of the Spearman rank correlation analysis (red, AF group; blue, non-AF group). (a) The correlations between plasma NT-proBNP level and rLMC score in the AF and non-AF groups. (b) The correlations between plasma NT-proBNP level and CTP ischemic volume in the AF and non-AF groups. (c) The correlations between plasma NT-proBNP level and CTP infarct core volume in the AF and non-AF groups. (d) The correlations between plasma NT-proBNP level and CTP ischemic penumbra volume in the AF and non-AF groups.

**Table 1:** Baseline characteristics of the patients and the single-factor analysis as stratified by the collateral status (*N* = 326).

Characteristics	Total population (*n* = 326)	AF group (*n* = 113)	Non-AF group (*n* = 213)	Test value	*P* value
Median age (IQR) (yr)	68.00 (56.00, 75.00)	74.00 (67.00, 80.00)	62.00 (53.00, 71.00)	5938.500	0.001
Male sex (no., %)	113 (34.7)	56 (27.2)	57 (47.5)	13.819^b^	0.001
TOAST (no., %)				245.220^b^	0.001
LAA	182 (55.8)	16 (14.2)	166 (77.9)		
CE	101 (31.0)	95 (84.1)	6 (2.8)		
SAO	27 (8.3)	1 (0.9)	26 (12.2)		
OC	8 (2.5)	1 (0.9)	7 (3.3)		
SUD	8 (2.5)	0 (0.0)	8 (3.8)		
Median SBP (IQR) (mmHg)	154.00 (135.00, 174.00)	150.00 (133.00, 168.00)	155.00 (138.50, 179.00)	10052.500	0.014
Median DBP (IQR) (mmHg)	87.50 (78.00, 100.00)	87.00 (77.00, 99.50)	89.00 (79.00, 101.00)	10830.500	0.137
Median glucose level on admission (IQR) (mmol/L)	6.87 (5.80, 9.00)	6.88 (5.94, 8.80)	6.86 (5.71, 9.11)	11853.000	0.823
Median NIHSS score on admission (IQR)	8 (3, 14)	12 (7, 16)	6 (3, 11)	7584.000	0.001
Median height (IQR) (m)	1.67 (1.60, 1.72)	1.63 (1.60, 1.70)	1.68 (1.60, 1.72)	9720.000	0.004
Median weight (IQR) (kg)	67 (60, 75)	65 (55, 74)	70 (60, 76)	9453.000	0.001
Median BMI (IQR) (kg/m^2^)	24.21 (22.04, 26.67)	23.44 (21.18, 27.02)	24.39 (22.43, 26.66)	10227.000	0.026
Median rLMC score (IQR)	18 (14, 20)	16 (13, 19)	19 (16, 20)	8365.000	0.001
Median CTP ischemic volume (IQR) (mL)	47.00 (5.75, 130.50)	64.00 (18.00, 162.00)	32.00 (0.00, 114.00)	9190.000	0.001
Median CTP infarct core volume (IQR) (mL)	4.00 (0.00, 20.25)	9.00 (1.00, 47.00)	2.00 (0.00, 14.00)	8891.500	0.001
Median CTP ischemic penumbra volume (IQR) (mL)	36.00 (4.00, 93.00)	56.00 (15.00, 102.00)	28.00 (0.00, 84.50)	9600.000	0.002
History of hypertension (no., %)	213 (65.3)	72 (63.7)	141 (66.2)	0.201^b^	0.654
History of diabetes mellitus (no., %)	77 (23.6)	22 (19.5)	55 (25.8)	1.652^b^	0.199
History of stroke (no., %)	37 (11.3)	16 (14.2)	21 (9.9)	1.357^b^	0.244
Family history of stroke (no., %)	68 (20.9)	22 (19.5)	46 (21.6)	0.202^b^	0.653
Smoking (no., %)	110 (33.7)	17 (15.0)	93 (43.7)	27.046^b^	0.001
Median NT-proBNP (IQR) (pg/mL)	157.40 (49.29, 901.60)	999.80 (554.20, 1695.00)	69.90 (36.25, 174.20)	2638.000	0.001
Median TnI (IQR) (pg/mL)	11.66 (7.45, 17.97)	13.79 (10.37, 23.65)	9.94 (6.59, 16.21)	8081.500	0.001
Median D-dimer (IQR) (ng/mL)	0.41 (0.23, 0.91)	0.76 (0.36, 1.38)	0.30 (0.22, 0.62)	7031.000	0.001
Mean PLT (SD) (^10^9^)	198.66 ± 58.77	176.64 ± 58.81	210.34 ± 55.43	-5.114^a^	0.436
Median INR (IQR)	1.04 (0.98, 1.10)	1.09 (1.04, 1.16)	1.02 (0.97, 1.08)	6714.000	0.001
Median FIB (IQR) (g/L)	3.10 (2.63, 3.63)	3.25 (2.62, 4.11)	3.04 (2.63, 3.58)	10484.000	0.056
Median APTT (IQR) (s)	32.75 (29.08, 35.93)	34.30 (30.65, 37.30)	32.30 (28.45, 35.30)	9442.000	0.001
Median Cr (IQR) (*μ*mol/L)	66.95 (57.00, 79.00)	66.90 (57.00, 79.00)	67.00 (57.00, 79.00)	11705.000	0.684
Median TG (IQR) (mmol/L)	1.21 (0.91, 1.63)	1.00 (0.74, 1.34)	1.31 (0.98, 1.81)	8013.500	0.001
Median TC (IQR) (mmol/L)	4.30 (3.68, 5.01)	3.87 (3.43, 4.52)	4.43 (3.85, 5.22)	8366.500	0.001
Median HDL-C (IQR) (mmol/L)	1.01 (0.86, 1.21)	1.01 (0.85, 1.26)	1.01 (0.86, 1.19)	11477.500	0.492
Mean LDL-C (SD) (mmol/L)	2.76 ± 0.91	2.51 ± 0.90	2.89 ± 0.88	-3.644^a^	0.847
Median ALB (IQR) (g/L)	40.75 (37.80, 43.60)	39.60 (36.60, 42.40)	41.30 (38.40, 44.05)	9501.500	0.002
Median Hcy (IQR) (*μ*mol/L)	11.00 (8.80, 13.80)	11.20 (9.80, 13.80)	10.50 (8.50, 13.95)	10733.000	0.123

Abbreviations: SBP: systolic blood pressure; DBP: diastolic blood pressure; NIHSS: National Institutes of Health Stroke Scale; BMI: body mass index; rLMC score: regional leptomeningeal collateral score. ^a^*t*-value. ^b^*χ*^2^ value. *P* value: intergroup difference.

**Table 2:** The Spearman rank correlation analysis of NT-proBNP level, rLMC score, and CTP status in the AF group (*n* = 113) and non-AF group (*n* = 213).

Variables	Total population (*n* = 326)		History of atrial fibrillation			
			Yes (*n* = 113)		No (*n* = 213)	
	*r*	*P* value	*r*	*P* value	*r*	*P* value
rLMC	-0.280	0.001	-0.156	0.022	-0.082	0.390
CTP ischemic volume	0.233	0.001	0.137	0.045	0.040	0.675
CTP infarct core volume	0.255	0.001	0.148	0.003	0.041	0.665
CTP ischemic penumbra volume	0.194	0.001	0.103	0.135	0.038	0.693

Abbreviation: rLMC score: regional leptomeningeal collateral score.

**Table 3:** Multivariate linear regression analysis with NIHSS score as a dependent variable in the AF group (*n* = 113).

Variables	Model 0			Model 1			Model 2		
	*B*	95% CI	*P*	*B*	95% CI	*P*	*B*	95% CI	*P*
Constant	16.188	11.678 to 20.698	<0.001	12.313	1.406 to 23.220	0.027	16.231	1.849 to 30.613	0.027
rLMC score	-0.459	-0.692 to -0.227	<0.001	-0.452	-0.690 to -0.214	<0.001	-0.430	-0.679 to -0.181	0.001
CTP ischemic penumbra volume	0.013	-0.006 to 0.033	0.177	0.014	-0.006 to 0.034	0.156	0.017	-0.005 to 0.038	0.127
NT-proBNP	0.001	0.000 to 0.002	0.004	0.001	0.000 to 0.002	0.004	0.001	0.000 to 0.002	0.002

Model 0: unadjusted; Model 1: adjusted for age, gender, and BMI; Model 2: adjusted for SBP, smoking status, TnI, D-dimer, INR, APTT, TG, TC, and ALB.

**Table 4:** Multivariate linear regression analysis with NIHSS score as a dependent variable in the non-AF group (*n* = 213).

Variables	Model 0			Model 1			Model 2		
	*B*	95% CI	*P*	*B*	95% CI	*P*	*B*	95% CI	*P*
Constant	16.475	11.970 to 20.980	<0.001	10.752	2.306 to 19.198	0.013	6.619	-5.287 to 18.525	0.274
rLMC score	-0.555	-0.790 to -0.320	<0.001	-0.533	-0.771 to -0.295	<0.001	-0.460	-0.701 to -0.219	<0.001
CTP ischemic penumbra volume	0.012	0.000 to 0.024	0.052	0.014	0.002 to 0.026	0.024	0.011	-0.001 to 0.023	0.078
NT-proBNP level	0.000	0.000 to 0.001	0.293	0.000	-0.001 to 0.001	0.675	0.000	-0.001 to 0.001	0.417

Model 0: unadjusted; Model 1: adjusted for age, gender, and BMI; Model 2: adjusted for SBP, smoking status, TnI, D-dimer, INR, APTT, TG, TC, and ALB.

## Data Availability

The datasets used and/or analyzed during the current study are available from the corresponding authors on reasonable request.

## Abbreviations

AF: Atrial fibrillation
BNP: B-type natriuretic peptide
CES: Cardioembolic stroke
CTP: Computed tomography perfusion
DWI: Diffusion-weighted imaging
ESUS: Embolic stroke of undetermined source
LAA: Large artery atherosclerosis
MRA: Magnetic resonance angiography
NIHSS: The National Institutes of Health Stroke Scale
NPs: Natriuretic peptides
NT-proBNP: N-terminal- (NT-) prohormone brain natriuretic peptide
rLMC: Regional leptomeningeal collateral.
